# Two-Stage Intelligent DarkNet-SqueezeNet Architecture-Based Framework for Multiclass Rice Grain Variety Identification

**DOI:** 10.1155/2022/1339469

**Published:** 2022-11-25

**Authors:** Maryam Fatima, Muhammad Attique Khan, Muhammad Sharif, Majed Alhaisoni, Abdullah Alqahtani, Usman Tariqe, Ye Jin Kim, Byoungchol Chang

**Affiliations:** ^1^Department of Computer Science, COMSATS University Islamabad, Wah Campus, Islamabad, Pakistan; ^2^Department of Computer Science, HITEC University, Taxila, Pakistan; ^3^Computer Sciences Department, College of Computer and Information Sciences, Princess Nourah Bint Abdulrahman University, Riyadh 11671, Saudi Arabia; ^4^College of Computer Engineering and Sciences, Prince Sattam Bin Abdulaziz University, Al-Kharj, Saudi Arabia; ^5^Department of Management Informatin Systems, CoBA, HITEC University, Taxila, Pakistan; ^6^Department of Computer Science, Hanyang University, Seoul 04763, Republic of Korea; ^7^Center for Computational Social Science, Hanyang University, Seoul 04763, Republic of Korea

## Abstract

Image processing is an important domain for identifying various crop varieties. Due to the large amount of rice and its varieties, manually detecting its qualities is a very tedious and time-consuming task. In this work, we propose a two-stage deep learning framework for detecting and classifying multiclass rice grain varieties. A series of steps is included in the proposed framework. The first step is to perform preprocessing on the selected dataset. The second step involves selecting and fine-tuning pretrained deep models from Darknet19 and SqueezeNet. Transfer learning is used to train the fine-tuned models on the selected dataset. The 50% sample images are employed for the training and rest 50% are used for the testing. Features are extracted and fused using a maximum correlation-based approach. This approach improved the classification performance; however, redundant information has also been included. An improved butterfly optimization algorithm (BOA) is proposed, in the next step, for the selection of the best features that are finally classified using several machine learning classifiers. The experimental process was conducted on selected rice datasets that include five types of rice varieties and achieves a maximum accuracy of 100% that was improved than the recent method. The average accuracy of the proposed method is obtained at 99.2%, through confidence interval-based analysis that shows the significance of this work.

## 1. Introduction

In the field of agriculture, rice is an unavoidable staple diet and the most used around the world [1]. In addition, it is the third most cultivated field in different areas, including China, East Asia, and the south [2, 3]. Approximately 90% of Asians prefer rice food, and their demand for rice increases day by day [4]. Myanmar is the largest rice exporter in the world and the sixth-largest rice-producing country [5]. Pakistan exports 8% of its rice to the world and the export rate is dependent on the quality of the rice [6]. To estimate the characteristic of a rice grain, various physical variables are utilized including shape, size, and texture, which are the most helpful feature to determine the quality of grain through image processing [7]. In other ways, it consumes much time in most procedures and despite that results were not better or more accurate, but image processing is a better option for identification of rice varieties [8]. The actual goal is to detect the rice grain quality within less time and cost.

Both physical and chemical methods are used for seed varieties of rice. In other words, destructive and nondestructive methods are also used for solving the rice problems [9]. These nondestructive methods are better as compared to destructive methods because nondestructive methods use the digital image processing (DIP) process, and now, people want to detect rice grain with less time and at cheaper rates. Stone, weed seeds, chaff, etc. are the main causes of damaging the seed quality [10]. Flatbed scanners are used for rice grading and inspection in which rice kernels, glass plate, and scanner head are used. The scanner detects the size, shape, density, and percentage of broken kernels [11]. Rice has different types. C4Raja rice [12], and kernel rice features depend on length, width, and perimeters [13]. Several rice types, such as Chenab Basmati, Kissan Basmati, Basmati 2000, KSK 133, KSK 434, Punjab Basmati, and PK 1121 aromatic, are mostly grown in Pakistan, are utilized for rice seed categorization, and have been gathered [14]. Some varieties are shown in Figure 1.

Rice grain quality and their varieties is an important factor in cultivation and import/export [16]. Manual labor and some machines work to solve these rice grain problems. Current machines are costly, so, to solve the quality problem, humans propose a machine vision algorithm [17] to identify the rice grain problem and solve them through classification method and based on images and videos, which is easy and fast in the detection of color, shape, and texture feature [18]. Different classification methods are used to classify rice into different groups [1]. On the contrary, automatic detection of the rice grain is a challenging task in the farming industry. Different applications of the technology are used for the automatic identification of rice grains [19]. To remove the impurities from the rice, different methods of DIP and probabilistic neural network (PNN) algorithms are utilized. To determine the grain's moisture content, machine learning (ML) techniques are applied [20]. Moreover, morphological methods are much important and play a significant part in determining the rice's quality.

In the field of agriculture, identifying and classifying a rice grain are one of the most interesting and demanding tasks. In the ongoing years, different machine learning-based approaches have been introduced. However, still, there are some gaps that need to be resolved in this area [21]. Several techniques have been introduced in the literature for rice variety detection and classification using computer vision and machine learning techniques [22]. Normally, they perform preprocessing techniques at the initial phase for better detection [23]. Robert Singh and Chaudhury [24] presented texture, wavelet, morphological, and color features which were used to classify the four different types of rice grain images that are taken using a 12-megapixel camera. The HSI channel has been used for image conversion and then these images (grayscale) converted into a binary image. Sethi et al. [6] used adaptive thresholding to convert the image into grayscale. Low pass and Gaussian filters are also used to smooth and denoise the image. Masking is used for highlighting the rice object. Histogram equalization (HE) is reviewing the gray level of the image, and image enhancement gives the idea that which techniques are applied to the grayscale and color image [25]. In the preprocessing process, the auto-align method is available to automatically align the arrangement and positioning of grain. The exact position around the grain used the contour method [26]. Wongruen [27] utilized four techniques based on segmentation such as fast K-means of Dixit, fuzzy C-means (FC), multilevel thresholding, and Otsu's multilevel thresholding (OMT). The OMT's and FC accuracy rates are 89.83% and 95.53%. Itharatet al. [28] used Khao Dawk MAli 105 dataset and applied global thresholding to segment the chalk area on images of rice. RiceNet-based segmentation has improved the quality of adhesive rice grain. We compare the result with region-based convolutional neural network (R-CNN) and give an 89.5% accuracy [29]. Bhupendra et al. [30] presented a deep learning architecture-based framework for rice grains' classification. They used several CNN models, and EfficientNetB0 successfully attained the accuracy of 98.32%. Moreover, classification is performed for several other fruit varieties by computer vision researchers such as date fruit [31], Pistachio Species [32], corn [33], and coffee beans [34].

In the abovementioned studies, the major problem is the appearance variation of several rice varieties. The similar shape, texture, irregularity, and rice width affect the rice segmentation accuracy. Furthermore, the incorrect segmentation step produced irrelevant features that later degrade the classification accuracy. Furthermore, in the classification phase, the presence of a few redundant and irrelevant features impacts the proposed framework's computational time (during the prediction process) and can decrease the classification accuracy. Another challenge is the selection of a classifier for final accuracy because several classifiers exist and many of them consumed a lot of time for the prediction process. Therefore, we proposed a two-stage framework for rice variety detection and classification. Our major contributions are as follows:

- We proposed a rice segmentation technique based on a color-based saliency map and thresholding
- Two pretrained deep models have been fine-tuned and have fused their information based on maximum correlation
- Best features are selected using an improved butterfly optimization algorithm

## 2. Proposed Methodology

In the proposed work, the main steps are the acquisition of a dataset, deep saliency-based rice segmentation, deep features extraction using pretrained models trained on the selected dataset, feature fusion, feature selection using an optimization technique, and finally classification through machine learning classifiers. The main flow of the proposed framework is illustrated in Figure 2. In Figure 2, it is noted that the saliency map is constructed that further processed in the form of a color map. Mathematically, each substep presented in this framework has been discussed below.

### 2.1. Saliency-Based Rice Segmentation

Segmentation is an important step in the domain of computer vision using plant application [35]. In this study, we introduced a saliency-based approach using Wang and Peng [36] technique. In this technique, we initially picked the superpixel image for the saliency method and select top, left, and right pixel for background seeds, the vector *B*_*v*_ = {*B*_1_, *B*_2_,… , *B*_*n*_}^*Z*^, and their values *B*_*p*_=1 and *B*_*p*_=0, this represents the labeled and unlabeled nodes, whereas *p* represents superpixel. The results of this method are shown in Figure 3. The background saliency is estimated as follows:

(1) $$\begin{array}{c} I_{v}={\left(K-\propto {\left(E^{J_{1}}\right)}^{-1}M^{J_{1}}\right)}^{-1}{\left(E^{J_{1}}\right)}^{-\left(1/2\right)}B_{v},\left(v=q,u,x\right)\text{,}\\ I_{b}\left(p\right)=1-norm\left(I_{q}\left(p\right).\;I_{u}\left(p\right).\;I_{x}\left(p\right)\right)\text{.} \end{array}$$

Diffusion-based compactness is defined as follows:

(2) $$\begin{array}{c} I_{f}\left(p\right)=1-norm\left(I_{v}\left(p\right)+I_{d}\left(p\right)\right)\text{,} \end{array}$$

where *I*_*v*_(*p*) is the spatial variance of superpixel and *I*_*d*_(*p*) is the spatial distance of superpixel. Later on, we combined the background saliency and compactness as follows:

(3) $$\begin{array}{c} I_{1}\left(p\right)=I_{b}\left(p\right)+I_{f}\left(p\right)\text{.} \end{array}$$

We jointly take into consideration the initial saliency values into the superior affinity network with the goal of creating a perspective of coarse-to-fine optimization to diffuse the first saliency map. Second, the robust affinity graph *M*^*J*_2_^ is computed as follows:

(4) $$\begin{array}{c} m_{ij}{\;}^{J_{2}}=m_{ij}{\;}^{J_{1}}+\left(m_{ij}{\;}^{y}\right)∙m_{ij}{\;}^{I_{f}}∙{\left(m_{ij}{\;}^{y}\right)}^{Z}\text{,} \end{array}$$

whereas *m*_*ij*_ ^*I*_*f*_^ is the affinity graph. We insert this graph into the manifold ranking objective function in order to achieve our goal of working the coarse-to-fine saliency result *I*_2_:

(5) $$\begin{array}{c} I_{v}={\left(K-\propto {\left(E^{J_{2}}\right)}^{-1}M^{J_{2}}\right)}^{-1}{\left(E^{J_{2}}\right)}^{-\left(1/2\right)}I_{2}\text{.} \end{array}$$

The lab color transformation is applied on *I*_2_, and the color mapped images are obtained which are later utilized for the training of pretrained deep learning models.

### 2.2. Pretrained Deep Models

In this work, two pretrained deep models have been employed for the training on rice dataset. The selected datasets are SqueezeNet and DarkNet19.

#### 2.2.1. SqueezeNet Model

A convolutional neural network of 18 layers deep is called SqueezeNet. The ImageNet database contains a pretrained version of the network that has been trained on almost a million photos.  Figure 4 shows SqueezeNet architecture and 3 CNNs highlighting the subset of layers. The SqueezeNet model is used for feature extraction. Final layer activation is dependent on the classification module, and these layers are complicated networks. There are two layers of the classification module: the global pooling layer and the convolutional layer. The remaining 2 layers are arbitrarily and pretrained on ImageNet. The detailed representation of the SqueezeNet model is shown in Table 1. Classification is performed on images through pretrained networks.

#### 2.2.2. DarkNet19

DarkNet19 is the convolutional neural network. We used the DarkNet19 model, in which 19 convolutional layers are known as DarkNet19. There are five max-pooling layers and 19 convolutional layers (CL) in DarkNet19, with several 1 × 1 CL to the minimum triangle parameters involving 3 × 3. We train the pretrained network by using a transfer learning technique that is applied to 75,000 images which provide the features of the network. In this stage, DarkNet19 was used to classify the images into 1000 classes, but we used only 5 classes for the results. Moreover, the image size of the input layer of DarkNet19 is 256 × 256. The view of the architecture neural network of DarkNet19 is shown in Figure 5. This network accepts the input of dimensional 244 × 244. The value of parameters and more details of the architecture neural network of DarkNet19 are shown in Table 2.

### 2.3. Transfer Learning

Transfer learning is used to improve the efficiency of the process and reduce the number of resources required. When elements of a pretrained machine learning model are reused in a new machine learning model, this is known as transfer learning. In transfer learning, we define feature vector and probability distribution as *A*={*f*_*v* _, *Pf*_*v*_)} and *f*_*v* _=*v*_1_, *v*_2_,…, *v*_*n*_, in which, the ground truth *G*=*g*_1_, *g*_2_,…, *g*_*n*_ and objective function *O*={*G*, *l*(*x*), whereas *l*(*x*) is unknown label class. *P*(*g|x*) is a probabilistic representation of the function. Transfer learning and learning rate are denoted as *T*_*o*_ and *L*_*o*_. *T*_*f*_ will be used to show the targeted function and the targeted output. The main goal of transfer learning is to improve the learning rate for predicting the targeted item using the recognition function (*l*(*x*)) depending upon the training learned from *T*_*o*_ and *T*_*f*_, where *T*_*o*_ ≠ *T*_*f*_ and *L*_*o*_ ≠ *T*_*f*_. Pattern recognition is improved via inductive transfer learning. When using inductive transfer learning, you will need an annotated database for fast training and testing. Visually, the process of transfer learning for the training of model on rice images is illustrated in Figure 6.

### 2.4. Features' Extraction and Fusion

Two feature vectors have been extracted from newly trained fine-tuned deep models. The first feature vector is extracted from SqueezeNet fine-tuned model and performed activation on second last feature layer. On this layer, 1024 features are extracted for each image. The second feature vector is extracted from DarkNet19 fine-tuned model and performed activation on second last convolutional layer. On this layer, 1000 features are extracted for each image. We fused both feature vectors using a proposed maximum correlation-based approach that combine the important information from both vectors.

We consider two feature vectors *F*_*v*1__ ^*Dar*^_, and *F*_*v*2_*Squ*, and fusion vector represented as *Fus*_*v*_. The dimension of these vectors is *R* × *N*, where *N* is represented as the number of images. Each one has a vector length of *R* × 1024 and *R* × 1000, respectively. The following formulation is performed to compute the correlation coefficient between two characteristics:

(6) $$\begin{array}{c} f\left(Dar\;,Squ\right)=\frac{COV\left(Dar\;,Squ\right)}{\sqrt{Var\left(Dar\right)}\;\sqrt{Var\left(Squ\right)}}\text{.} \end{array}$$

The range of these values, *Dar* and *Squ*, lies between (−1 and 1). -1 stands for weak correlation, and 1 stands for strong correlation. The equation of maximum correlation vector is defined as follows:

(7) $$\begin{array}{c} CV\left(Dar\;,Squ\right)=\varphi \;f\left(m_{1}\left(Dar\right),m_{2}\left(Squ\right)\right) \end{array}$$

where *φ* denotes the supremum of the overall Borel functions [37], *Squ*: *ω*⟶*ω* is located between (0 and 1), and *CV*(*Dar* , *Squ*) is the maximum correlation. If the correlation is close to 1, then we drop it; if it is 0, then we discard both features through fused vector. Based on this formulation, a fusion vector is obtained having dimension *N* × 931 that later processes in the optimization algorithm for the best feature selection.

### 2.5. Improved Butterfly Optimization Algorithm-Based Feature Selection

A technique for reducing the input variable to your model is feature selection, which involves removing noise and using just useful data. It involves selecting the best characteristics for your machine learning model in accordance with the kind of issue you are seeking to tackle automatically. The butterfly optimization algorithm (BOA) is the metaheuristic algorithm [38]. Metaheuristic is a relatively new type of optimization algorithm that is used to find the best solution and is influenced by the food investigating behavior of butterflies. Initially, the physical stimulus intensity work on the perceived intensity of the fragrance (*f*) is defined as follows:

(8) $$\begin{array}{c} f={eL}^{d}\text{,} \end{array}$$

where *e*, *d*, and *L* are sensory mandatory, stimulus intensity, and power exponent that depends on modality. The best global butterfly position can be represented as

(9) $$\begin{array}{c} P_{j}^{m+1}=P_{j}^{m}+\left({rn}^{2}\times b_{p}-P_{j}^{m}\right)\times f_{j}\text{,} \end{array}$$

where *P*_*j*_^*m*^ is *j*^*th*^ butterfly position at time *m* and *rn* is the random number [0,1]. *f*_*j*_ is the fragrance of *jth* butterfly and *b*_*p*_ is the best current position. The local walk is defined as

(10) $$\begin{array}{c} P_{j}^{m+1}=P_{j}^{m}+\left({rn}^{2}\times P_{k}^{m}-P_{l}^{m}\right)\times f_{j}\text{,} \end{array}$$

where *rn* is the random number of between [0,1] and *P*_*k*_^*m*^ and *P*_*l*_^*m*^ are used for *kth* and *lth* butterfly's position. In the following step, the selected features based on the above equation are passed to the cross-entropy (CE) function. CE is used for the global search for butterfly's movement. The following is an optimization problem:

(11) $$\begin{array}{c} {\;}_{z\in Z}^{\mathrm{Min}}R\left(z\right)\text{,} \end{array}$$

where *Z* defined the final states and *R* is the real value performance function *Z*. An auxiliary problem and probability distribution estimation problem are described as follows:

(12) $$\begin{array}{c} L\left(\gamma \right)=P_{m}\left(S\left(R\right)\leq \gamma =E_{o}\left[F_{\left\{S\left(R\right)\leq \gamma \right\}}\right]\right.\text{,} \end{array}$$

where *P*_*m*_ is the probability measure, *S*(*R*) is the random state, *E*_*o*_ is the expected operator, *γ* show the thresholding parameter, and *F* shows the indicator function (the value of F is 1 if *S*(*R*) ≤ *γ*, 0). In the CE method, the significance sampling methodology is employed to lower the sample size. As a result, the equation can be rewritten like this

(13) $$\begin{array}{c} L\left(\gamma \right)=\frac{1}{n}\overset{n}{\underset{j}{\sum }}FS\left(R\right)\leq \gamma \frac{e\left(y_{i};a\right)}{h\left(y_{i}\right)}\text{,} \end{array}$$

where *e*(*y*_*i*_; *a*) represents the random sample and *h*(*y*_*i*_) represents optimal density that can be discovered by reducing the Kullback–Leibler divergence:

(14) $$\begin{array}{c} \begin{array}{c} \min\\ a \end{array}\frac{1}{n}\overset{n}{\underset{j}{\sum }}FS\left(R\right)\leq \gamma In\;e\left(y_{i};a\right)\text{.} \end{array}$$

Hence, the final optimization can be done as follows:

(15) $$\begin{array}{c} a_{k+1}^{*}={\propto a}^{+}+\left(1-\propto \right)a_{k}^{*}\text{,} \end{array}$$

whereas the smoothing parameter is 0≤∝≤1. This improved algorithm continues until the number of iterations is not completed. In this work, the numbers of iterations are 200. At the end, we obtained a feature vector of dimensional *N* × 522 which was finally classified using machine learning classifiers.

## 3. Results and Discussion

### 3.1. Dataset

In this work, we utilized a publically available rice dataset that include five types of rice varieties such as (a) Khazar, (b) Gharib, (c) Ghasrdashti, (d) Gerdeh, and (e) Mohammadi [39]. A sample image is shown in Figure 1. This dataset consists of total 75,000 images and each class consists of 15,000 images (https://www.kaggle.com/datasets/muratkokludataset/rice-image-dataset). We employed 50% of the images from each class for training and rest for testing.

### 3.2. Experimental Setup

The experimental process of the proposed method is conducted on publically available rice imaging dataset [39], as discussed under Section 3.1. We performed the 50 : 50 approach for both training and testing, whereas the cross-validation value is 10. Four different experiments have been performed for the detailed analysis of the proposed method. In the first experiment, the DarkNet19 model is used after applying deep saliency-based segmentation on the datasets and fed to the classifier. In the second experiment, we train the dataset through the SqueezeNet model and fed it to the classifier. In the third experiment, we applied feature fusion both the first and second models fused the features and fed them to the classifier. At the end, the best value of features is selected through improved butterfly optimization. Several classifiers have been opted for the classification, whereas the performance of each classifier is computed based on recall rate, precision rate, *F*1 score, and accuracy. Moreover, the computational time is noted during the testing process. The entire proposed method is implemented on MATLAB2022a using Desktop Computer with 16 GB of RAM and 6 GB NVIDIA RTX graphics card.

### 3.3. Experiment 1: DarkNet19 Features

In experiment 1, segmentation is performed on the selected dataset through the proposed approach. After segmentation, we train the fine-tuned DarkNet19 model and extract deep features. On this model, 1024 features have been extracted. Ten different classification methods have been opted and performed classification. The testing accuracy on multiple classifiers is depicted in Table 3. In this table, the accuracy of quadratic SVM is 98.4%, which is better compared to other well-known classification methods such as linear SVM, weight KNN, cosine KNN, linear discriminant, and five types of neural networks. The second highest accuracy of 98.3% was obtained on linear SVM and linear discriminant classifiers. The linear discriminants have taken less time as compared to other classifiers. The performance measure of quadratic SVM is also illustrated by a confusion matrix (CM) shown in Figure 7.

### 3.4. Experiment 2: SqueezeNet Features

In experiment 2, SequeezeNet testing features have been extracted and classification has been performed. From this model, 1000 features are extracted. Ten classifiers have been utilized for the classification results and obtained the maximum accuracy of 99.5% by quadratic SVM, as presented in Table 4. The other classifiers also give better accuracy, but the maximum accuracy is obtained on quadratic SVM. The computational time is also noted for all classifiers, and it is observed that the linear discriminant consumes less time than the rest of the classifiers. Moreover, the confusion matrix of quadratic SVM is also provided as illustrated in Figure 8.

### 3.5. Experiment 3: Feature Fusion

In the third experiment, extracted deep learning features are fused using the proposed maximum correlation-based approach. Similar to experiment 1 and experiment 2, ten different classification methods have been utilized, and the results are presented in Table 5. In this table, it is noted that the accuracy is improved after the fusion process, whereas the time is slightly decreased. The wide neural network better performed than the rest of the classifiers as the obtained accuracy is 100% and computational time is 139.86 (sec). Compared to experiment 1 and experiment 2, all classifiers performed better after the fusion process. Moreover, the confusion matrix is also provided as illustrated in Figure 9. In this figure, it is clearly observed that each class correct prediction rate is above 99%.

### 3.6. Experiment 4: Best Selected Features

In experiment 4, the best features are selected using the proposed improved butterfly optimization algorithm. The total 522 features are selected after employing the proposed optimization algorithm. Results of this experiment are given in Table 6. The best noted accuracy of 100% was achieved by Cubic SVM, whereas the recall rate is 99.98, precision rate is 99.96, and *F*1 score is 99.96%, respectively. The other classifiers also obtained better accuracy and consumed less time than the previous experiments. The confusion matrix of quadratic SVM is also given as illustrated in Figure 10.

### 3.7. Analysis and Comparison

In this section, a detailed analysis of the proposed system is conducted based on numerical values and some visual plots. The proposed method was evaluated on a publicly available dataset including five classes as illustrated in Figure 1. The proposed method includes some important steps such as rice segmentation, deep learning feature extraction, fusion of deep features using the proposed approach, and selection of best features using improved butterfly optimization; the main flow is given in Figure 2. The proposed segmentation technique clearly highlights the rice region shown in Figure 3 which is later utilized for the training of deep models. The results of each step are computed as given in Tables 3–6. Moreover, the confusion matrix of step is illustrated in Figures 7–10. Based on the results, it is clearly observed that the fusion process reduces the computational time that further reduces after the best feature selection. Moreover, we conducted a comparison of the proposed method with several other neural networks as illustrated in Figure 11. Based on this figure, it is clearly shown that the proposed fusion and selection methods give better accuracy.

Finally, a comparison is conducted with recent techniques on rice_image_dataset, as presented in Table 7. Koklu et al. [39] used a rice image dataset and applied three classification methods. The classifier ANN, DNN, and CNN and their results are 99.87%, 99.95%, and 100%, respectively. Cinar and Koklu [40] used the same dataset and achieved maximum accuracy of 99.9%. In [41], authors presented a deep learning-based framework for rice variety classification and obtained accuracy of 98.2%. In [42], authors presented a computerized method and obtained 93.04% accuracy. The proposed method achieved the maximum 100% accuracy with minimum computational time.

## 4. Conclusion

In this study, we proposed an automated deep learning-based framework for rice segmentation and variety classification. The proposed framework includes several critical steps. For better visualization, the segmentation step localized the rice region and mapped color. The main goal of this step is to provide better images for deep learning model training. Two pretrained deep models extract features from segmented mapped images. The extracted features are fused using the proposed maximum correlation-based technique. This step reduced the number of features and selected only the most important ones for the fused matrix. However, it should be noted that, during the experimental process, some redundant features are also added to the fused matrix, which does not affect accuracy but increases computational time. As a result, we proposed an improved butterfly optimization algorithm that not only maintains accuracy but also reduces testing time. The selection of important features during the fusion process is the main limitation of this work using the static threshold value. In the future, the fusion process will be optimized for less computational time by employing new techniques. Moreover, in the future, plant and rice disease detection and classification problems will be considered [43–47].

## Figures and Tables

**Figure 1:** Rice varieties: (a) Khazar, (b) Gharib, (c) Ghasrdashti, (d) Gerdeh, and (e) Mohammadi [15].

**Figure 2:** Proposed deep learning and optimization-based framework of rice variety classification.

**Figure 3:** (a) Original data. (b) Proposed saliency-based segmented images.

**Figure 4:** SqueezeNet architecture.

**Figure 5:** Architecture of DarkNet19.

**Figure 6:** Deep transfer learning.

**Figure 7:** Confusion matrix of quadratic SVM (experiment 1).

**Figure 8:** Confusion matrix of quadratic SVM (experiment 2).

**Figure 9:** Confusion matrix of wide neural network (experiment 3).

**Figure 10:** Confusion matrix of quadratic SVM (experiment 4).

**Figure 11:** Comparison of the proposed method with other neural networks.

**Table 1:** Description of SqueezeNet architecture.

Layer name/type	Output size	Filter size/stride(if not a fire layer)	Depth	S1 × 1 (#1 × 1 squeeze)	e1 × 1 (#1 × 1 expand)	e3 × 3 (#3 × 3expand)
Input image	224 × 224					
Conv1	111 × 111 × 96	7 × 7/ (x96)	1			
Maxpool1	55 × 55 × 96	3 × 3/2	0			
Fire 2	55 × 55 × 128		2	16	64	64
Fire 3	55 × 55 × 128		2	16	64	64
Fire 4	55 × 55 × 256		2	32	128	128
Maxpool4	27 × 27 × 256	3 × 3/2	0			
Fire 5	27 × 27 × 256		2	32	128	128
Fire 6	27 × 27 × 384		2	48	192	192
Fire 7	27 × 27 × 384		2	48	192	192
Fire 8	27 × 27 × 512		2	64	256	256
Maxpool8	13 × 12 × 512	3 × 3/2	0			
Fire 9	13 × 13 × 512		2	64	256	256
Conv10	13 × 13 × 5	1 × 1/1 (×5)	1			
Avgpool10	1 × 1 × 5	13 × 13/1	0			

**Table 2:** Description of DarkNet19 architecture.

Type	Filters	Size/stride	Output
Convolutional	34	3 × 3	224 × 2 24
Maxpool		2 × 2/2	112 × 112
Convolutional	64	3 × 3	112 × 112
Maxpool		2 × 2/2	56 × 56
Convolutional	128	3 × 3	56 × 56
Convolutional	64	1 × 1	56 × 56
Convolutional	128	3 × 3	56 × 56
Maxpool		2 × 2/2	28 × 28
Convolutional	256	3 × 3	28 × 28
Convolutional	128	1 × 1	28 × 28
Convolutional	256	3 × 3	28 × 28
Maxpool		2 × 2/2	14 × 14
Convolutional	512	3 × 3	14 × 14
Convolutional	256	1 × 1	14 × 14
Convolutional	512	3 × 3	14 × 14
Convolutional	256	1 × 1	14 × 14
Convolutional	512	3 × 3	14 × 14
Maxpool		2 × 2/2	7 × 7
Convolutional	1024	3 × 3	7 × 7
Convolutional	512	1 × 1	7 × 7
Convolutional	1024	3 × 3	7 × 7
Convolutional	512	1 × 1	7 × 7
Convolutional	1024	3 × 3	7 × 7
**Convolutional**	**5**	**1 × 1**	**7 × 7**
New_softmax		Global	5

**Table 3:** Classification results of the DarkNet19 model (experiment 1).

Classifier (%)	Recall (%)	Precision (%)	*F*1 score (%)	FNR (%)	Accuracy (%)	Time (sec)
Linear SVM	98.28	98.3	98.29	1.72	98.3	277.71
**Quadratic SVM**	98.36	98.38	98.37	1.64	**98.4**	291.46
Weight KNN	98.22	98.2	98.21	1.78	98.2	1444.8
Cosine KNN	98.2	98.22	98.21	1.8	98.2	1781.5
Linear discriminant	98.26	98.28	98.27	1.74	98.3	**73.55**
Medium neural network	97.86	97.88	97.87	2.14	97.9	1203.3
Narrow neural network	97.76	97.74	97.75	2.24	97.8	1943.7
Wide neural network	97.9	97.88	97.89	2.1	97.9	1699.8
Bilayered neural network	97.82	97.84	97.83	2.18	97.8	2330.2
Trilayered neural network	97.82	97.88	97.85	2.18	97.8	1922.5

**Table 4:** Classification results of the SqueezeNet model (experiment 2).

Classifier (%)	Recall (%)	Sensitive (%)	*F*1 score (%)	FNR (%)	Accuracy (%)	Time (sec)
Linear SVM	99.22	99.24	99.23	0.78	99.2	301.74
**Quadratic SVM**	99.46	99.46	99.4	0.54	**99.5**	304.67
Weight KNN	98.58	98.44	98.51	1.42	98.6	362.9
Cosine KNN	97.9	97.94	97.92	2.1	97.9	387.4
Linear discriminant	99.32	99.32	99.32	0.68	99.3	**72.783**
Medium neural network	99.42	99.42	99.42	0.58	99.4	178.13
Narrow neural network	99.38	99.38	99.38	0.62	99.4	244.41
Wide neural network	99.41	99.4	99.41	0.58	99.4	249.99
Bilayered neural network	99.36	99.36	99.36	0.64	99.4	336.25
Trilayered neural network	99.37	99.38	99.37	0.64	99.4	458.32

**Table 5:** Classification results of fusion data (experiment 3).

Classifier (%)	Recall (%)	Sensitive (%)	*F*1 score (%)	FNR (%)	Accuracy (%)	Time (sec)
Linear SVM	99.96	99.94	99.95	0.04	99.9	275.3
Quadratic SVM	99.96	99.96	99.96	0.04	100	221.12
Weight KNN	99.88	99.7	99.79	0.12	99.9	133.5
Cosine KNN	99.86	99.88	99.87	0.14	99.9	146.3
Linear discriminant	99.76	99.76	99.76	0.24	99.7	143.63
Medium neural network	99.94	99.94	99.94	0.06	99.9	223.75
Narrow neural network	99.92	99.96	99.94	0.08	99.9	209.29
**Wide neural network**	99.96	99.96	99.96	0.04	**100**	**139.86**
Bilayered neural network	99.94	99.96	99.95	0.06	99.9	204.31
Trilayered neural network	99.9	99.92	99.91	0.1	99.9	229.86

**Table 6:** Classification result after proposed optimization algorithm (experiment 4).

Classifier	Recall (%)	Precision rate (%)	*F*1 score (%)	FNR (%)	Accuracy (%)	Time (sec)
Linear SVM	99.4	99.94	99.94	0.6	99.9	108.64
**Quadratic SVM**	99.98	99.96	99.96	0.02	**100**	142.31
Weight KNN	99.88	99.9	99.89	0.12	99.9	179.7
Cosine KNN	99.86	99.86	99.86	0.14	99.9	51.49
Linear discriminant	99.68	99.7	99.69	0.32	99.7	53.094
Medium neural network	99.74	99.74	99.74	0.26	99.9	63.839
Narrow neural network	99.9	99.7	99.81	0.1	99.9	71.045
Wide neural network	99.92	99.96	99.94	0.08	99.9	43.207
Bilayered neural network	99.94	99.92	99.93	0.06	99.9	86.704
Trilayered neural network	99.94	99.92	99.93	0.06	99.9	97.371

**Table 7:** Comparison results of others' work.

References	Year	Dataset	Accuracy (%)	
[39]	2021	Rice_image_dataset	ANN	99.87
			DNN	99.95
			CNN	100

[40]	2022	Rice_image_dataset	Logistic regression	99.25
			Multiperceptron	99.9
			Classification	97.4

[41]	2022	Rice_Image_dataset	Classification	98.2
[42]	2022	Rice dataset	Classification	93.04
Proposed	**2022**	**Rice_image_dataset**	**Linear SVM**	**99.9**
			**Quadratic SVM**	**100**
			**Weight CNN**	**99.9**
			**Cosine CNN**	**99.9**
			**Linear discriminant**	**99.7**
			**Medium NN**	**99.9**
			**Narrow NN**	**99.9**
			**Wide NN**	**99.9**
			**Bilayered NN**	**99.9**
			**Trilayered NN**	**99.9**

## Data Availability

The publicly available dataset has been used in this work for the experimental process (https://www.kaggle.com/datasets/muratkokludataset/rice-image-dataset).
